# Regulation of Nuclear Factor-kappaB Function by *O*-GlcNAcylation in Inflammation and Cancer

**DOI:** 10.3389/fcell.2021.751761

**Published:** 2021-10-15

**Authors:** Angela Rose Liu, Parameswaran Ramakrishnan

**Affiliations:** ^1^Department of Pathology, Case Western Reserve University, Cleveland, OH, United States; ^2^The Case Comprehensive Cancer Center, Case Western Reserve University, Cleveland, OH, United States; ^3^Department of Biochemistry, School of Medicine, Case Western Reserve University, Cleveland, OH, United States

**Keywords:** inflammation, cancer, posttranslational modifications (PTMs), *O*-GlcNAcylation, NF-kappaB (NF-κB), leukemia, hexosamine biosynthetic pathway

## Abstract

Nuclear factor-kappaB (NF-κB) is a pleiotropic, evolutionarily conserved transcription factor family that plays a central role in regulating immune responses, inflammation, cell survival, and apoptosis. Great strides have been made in the past three decades to understand the role of NF-κB in physiological and pathological conditions. Carcinogenesis is associated with constitutive activation of NF-κB that promotes tumor cell proliferation, angiogenesis, and apoptosis evasion. NF-κB is ubiquitously expressed, however, its activity is under tight regulation by inhibitors of the pathway and through multiple posttranslational modifications. *O*-GlcNAcylation is a dynamic posttranslational modification that controls NF-κB-dependent transactivation. *O*-GlcNAcylation acts as a nutrient-dependent rheostat of cellular signaling. Increased uptake of glucose and glutamine by cancer cells enhances NF-κB *O*-GlcNAcylation. Growing evidence indicates that *O*-GlcNAcylation of NF-κB is a key molecular mechanism that regulates cancer cell proliferation, survival and metastasis and acts as link between inflammation and cancer. In this review, we are attempting to summarize the current understanding of the cohesive role of NF-κB O-GlcNAcylation in inflammation and cancer.

## Introduction

The nuclear factor kappaB (NF-κB) family is a highly conserved group of master transcription factors critical in regulating cellular functions including cell survival, proliferation, differentiation, apoptosis, and immune response. NF-κB is composed of five subunits: p65 (RelA), RelB, c-Rel (Rel), p50/p105 (NF-κB1), and p52/p100 (NF-κB2) which exists as homo and heterodimers bound to the of inhibitor of kappaB (IκB) proteins (Hayden and Ghosh, 2011). NF-κB exists as preformed proteins, and its functional regulation primarily occurs through stimulus-dependent posttranslational modifications (PTMs) including phosphorylation, methylation, ubiquitination, acetylation, nitrosylation, sumoylation, and *O*-linked β-*N*-acetylglucosamine glycosylation (*O*-GlcNAcylation). Extensive crosstalk between PTMs (e.g., phosphorylation/*O*-GlcNAcylation) also regulates the function of NF-κB (Liu et al., 2004; Wang et al., 2007, 2008; Hart et al., 2011).

*O*-GlcNAcylation has garnered considerable interest in physiology and pathology since its discovery (Torres and Hart, 1984). *O*-GlcNAcylation is a posttranslational enzymatic addition of an N-acetylglucosamine (GlcNAc) to the oxygen atom of a serine, threonine, or tyrosine residue on intracellular proteins through a β-*O*-glycosidic linkage. In contrast to the abundance of kinases and phosphatases controlling phosphorylation (Ardito et al., 2017), *O*-GlcNAc cycling is controlled solely by the reciprocal activities of *O*-GlcNAc transferase (OGT) and *O*-GlcNAcase (OGA), which adds and removes *O*-GlcNAc from proteins, respectively. *Ogt* deficiency results in embryonic lethality (Shafi et al., 2000) and *Oga* deficiency affects embryonic development leading to neonatal lethality (Yang et al., 2012). Conditional deletion of *Ogt* showed the requirement of *O*-GlcNAcylation in T cell and fibroblast survival (O’Donnell et al., 2004) while conditional deletion of *Oga* in hematopoietic stem cells showed that *O*-GlcNAcylation cycling is essential in early thymocyte development (Abramowitz et al., 2019). Increased *O*-GlcNAcylation also blocks RANKL-induced p65 phosphorylation and suppresses osteoclastogenesis (Takeuchi et al., 2016). In addition to development, *O*-GlcNAcylation regulates a plethora of cellular functions, including cell survival, apoptosis, cell cycle, cell proliferation, stress response, and immune response, by controlling transcription, translation, and protein stability. A large number of *O*-GlcNAcylated proteins are involved in transcription regulation, including transcription factors such as NF-κB (Hart et al., 2007; Li et al., 2019). Exposure to high glucose or glucosamine induces NF-κB *O*-GlcNAcylation and increases NF-κB-dependent gene expression (James et al., 2002). NF-κB *O*-GlcNAcylation occurs via direct binding to OGT (Golks et al., 2007). Multiple sites of NF-κB p65 *O*-GlcNAcylation were later identified to have specific functional roles (Yang et al., 2008; Allison et al., 2012; Ma et al., 2017). We discovered that, unlike p65 with multiple *O*-GlcNAcylation sites, NF-κB c-Rel has a single *O*-GlcNAcylation site at Ser-350. Approximately 5% of c-Rel is *O*-GlcNAcylated under physiological glucose conditions (5 mM), while 25% of c-Rel is *O*-GlcNAcylated under hyperglycemic conditions (30 mM) (Ramakrishnan et al., 2013). The stoichiometry of p65 *O*-GlcNAcylation has yet to be defined. *O*-GlcNAcylation also modifies other proteins within the NF-κB pathway. Ser-733 *O*-GlcNAcylation of IKK2 is essential for its catalytic activity (Kawauchi et al., 2009). Similarly, TAB3 and TAB1 are *O*-GlcNAcylated at Ser-408, and Ser-395, respectively (Pathak et al., 2012; Tao et al., 2016; Figure 1).

**FIGURE 1:** Overview of *O*-GlcNAcylation sites and other posttranslational modifications in the nuclear factor-kappaB (NF-κB) pathway proteins. Shown are the principle structural motifs and posttranslational modification sites of p65, c-Rel, IKK2, TAB1, and TAB3. RHD, rel homology domain; TAD, transactivation domain; KD, kinase domain; LZ, leucine zipper; HLH: helix-loop-helix domain, NBD, Nemo-binding domain; PD, pseudophosphatase domain, TBD, TAK1 binding domain; CUE, coupling of ubiquitin conjugation to endoplasmic reticulum degradation; NZF, Npl4 zinc finger. *Activity has been shown to have crosstalk with *O*-GlcNAcylation; **Site specific acetylation but not methylation at this site has been shown to be related to *O*-GlcNAcylation.

*O*-GlcNAcylation is regulated by nutrient availability. Influxes of glucose and its metabolic products activate the hexosamine biosynthetic pathway (HBP) and enhance *O*-GlcNAcylation (Hanover et al., 2010; Chiaradonna et al., 2018). Cancer cells favor glycolysis and lactate fermentation for their survival and proliferation, a biological phenomenon called the Warburg effect (Liberti and Locasale, 2016). Cancer cells also consume excess glutamine to sustain protein synthesis (Rajagopalan and DeBerardinis, 2011). An increase of total protein *O*-GlcNAcylation due to the influx of glucose and glucosamine is a typical characteristic in cancer cells (Ma and Vosseller, 2014; Ferrer et al., 2016). Constitutively overactive NF-κB is also common in both solid and hematological cancers (Karin et al., 2002; Imbert and Peyron, 2017), with altered NF-κB expression associated with worse patient outcomes (Wu et al., 2015). In turn, enhanced NF-κB *O*-GlcNAcylation alters the homeostatic regulation of NF-κB-dependent transcription in cancer cells. This review summarizes the current knowledge on NF-κB *O*-GlcNAcylation as a molecular mechanism that connects inflammation and cancer, and discusses its potential therapeutic implications and future perspectives.

## Nuclear Factor-Kappab *O*-Glcnacylation in Solid Cancer

Elevated global protein *O*-GlcNAcylation is a common finding in several solid cancers including breast (Caldwell et al., 2010; Krześlak et al., 2012), prostate (Lynch et al., 2012), colorectal (Mi et al., 2011), and liver (Zhu et al., 2012). These cancers are also associated with dysregulated NF-κB function, which contributes to tumorigenesis (Xia et al., 2014). There have been many studies separately identifying the importance of NF-κB signaling and *O*-GlcNAcylation in tumor development, however, few have linked them together directly. Suppression of IKK2 significantly decreases tumor development in colitis-associated colon cancer (Greten et al., 2004). Separately, inhibition of bacterial (He et al., 2020) and murine (Yang et al., 2015) colonic *O*-GlcNAcylation is protective against colitis development possibly due to the disruption of p65 activation, which may also involve IKK2 *O*-GlcNAcylation. NF-κB signaling (Meylan et al., 2009; Bassères et al., 2010) and global *O*-GlcNAcylation (Taparra et al., 2018) are both required for the development of KRAS-induced lung cancer in mouse models. NF-κB activity facilitates the cell cycle transition from the G1 to S phase through antagonizing p53 and upregulating cyclin D1 gene expression (Chen et al., 2001) which is correlated with decreased *O*-GlcNAcylation (Wang et al., 2010; Drougat et al., 2012). Interestingly, there are specific instances in which NF-κB acts as a tumor suppressor. NF-κB inhibition in hepatocytes via IKK2-targeted deletion promotes hepatocarcinogenesis (Maeda et al., 2005). Separately, enhanced *O*-GlcNAcylation is seen in patients who suffered from tumor recurrence following liver transplantation. Taken together, this indicates that enhanced *O*-GlcNAcylation may inhibit NF-κB activation in hepatocytes to promote hepatocarcinogenesis. More research must be completed to specifically learn the tissue specific activating or inhibitory roles of NF-κB *O*-GlcNAcylation.

The existence of enhanced NF-κB activation and increased *O*-GlcNAcylation in several cancers beg the question: is site specific NF-κB *O*-GlcNAcylation involved in cancer pathogenesis? Several studies justify this possibility (Table 1). Enhancement of p65 *O*-GlcNAcylation is associated with the upregulation of CXCR4 expression in metastasized cervical cancer cells in the lung (Ali et al., 2017) suggesting that enhanced p65 *O*-GlcNAcylation during cancer may increase the metastatic potential of tumor cells. Furthermore, enhanced *O*-GlcNAcylation upregulates expression of matrix-metalloproteinases via increased p65 nuclear translocation resulting in an NF-κB *O*-GlcNAcylation-dependent increase in cholangiocarcinoma cell migration and invasion (Phoomak et al., 2016). Enhanced p65 nuclear translocation can be correlated with the decreased interaction between Thr-352 *O*-GlcNAcylated p65 and its physiological repressor, IκBα (Yang et al., 2008). *O*-GlcNAcylation at Thr-352, but not Thr-322, is required for p65 transcriptional activity (Yang et al., 2008), but *O*-GlcNAcylation at both sites is required for the anchorage of pancreatic ductal adenocarcinoma cells *in vitro* (Ma et al., 2013; Figure 1). Thus, enhanced site-specific p65 *O*-GlcNAcylation may contribute to the ability of tumor cells to invade and metastasize: a key hallmark of cancer. It is unclear whether or not *O*-GlcNAcylated p65 regulates gene expression differentially across various tissue types, and if it causes altered nuclear translocation, differential dimerization with other proteins, modulation of p65-DNA binding, or a combination of several functions.

**TABLE 1:** List of known *O*-GlcNAcylation sites and functions in the nuclear factor-kappaB (NF-κB) pathway proteins.

Aside from p65, *O*-GlcNAcylation of other NF-κB signaling proteins can also be involved in solid tumor pathogenesis. TAB3 *O*-GlcNAcylation promotes triple negative breast cancer cell migration and invasion, and is correlated with worse patient outcomes (Tao et al., 2016). Enhanced *O*-GlcNAcylation of IKK2 induces NF-κB signaling (Kawauchi et al., 2009), and increased IKK2 expression is essential for cell viability in prostate cancer (Pflueger et al., 2011). This suggests that *O*-GlcNAcylation may regulate IKK2 function to create a cell survival advantage. More research is needed to specifically address the mechanistic role of *O*-GlcNAcylation of NF-κB pathway proteins in carcinogenesis and cancer progression.

## Nuclear Factor-Kappab *O*-Glcnacylation in Hematological Cancers

The role of NF-κB *O*-GlcNAcylation in hematological cancers is largely unknown. Enhanced *O*-GlcNAcylation promotes multiple myeloma cell survival by increasing proteasome biogenesis and function to contribute to proteasomal inhibitor drug resistance (Sekine et al., 2018; Hashimoto et al., 2020). Heightened proteasome function may possibly result in an increase of IκBα degradation and subsequently enhance NF-κB activation in multiple myeloma, as seen in pancreatic cancer cells (Ma et al., 2013). Thus, elevated *O*-GlcNAcylation may worsen multiple myeloma patient outcomes through enhanced NF-κB activation causing diminished treatment efficacy. The reported function of global *O*-GlcNAcylation in leukemia is mixed. Enhanced *O*-GlcNAcylation is associated with chronic lymphocytic (Shi et al., 2010) and pre-B acute lymphocytic (Zhang et al., 2017) leukemia pathogenesis, and is accompanied with constitutive NF-κB activity due to the persistent activation of IκB kinases (Kordes et al., 2000; Takaesu et al., 2000; Bichi et al., 2002). Enhanced *O*-GlcNAcylation (Asthana et al., 2018) and aberrant NF-κB activity (Guzman et al., 2001) also occur in acute myeloid leukemia, and pharmacological inhibition of *O*-GlcNAcylation is able to induce the differentiation and apoptosis of AML cells (Asthana et al., 2018), However, contrasting studies have shown that enhanced *O*-GlcNAcylation via an increase of OGT protein expression via hypomethylation of its 5’ UTR promoter region using dronabinol also induces acute myeloid leukemic cell apoptosis and releases the differentiation blockage of acute myeloid leukemic blasts (Kampa-Schittenhelm et al., 2020). This contrasting data can potentially be explained due to the usage of a mouse xenograft model versus human patient samples with specific molecular mutations. Dronabinol also acts as an unselective epigenetic modifier, and while its effect on OGT was identified as a key regulator in instigating leukemia cell apoptosis and differentiation, it is possible that cross talk or contribution from other proteins is occurring. It is also notable that neither of these reports identified specific *O*-GlcNAcylated proteins that regulate this phenomenon seen in AML cells. Additional studies on NF-κB-specific *O*-GlcNAcylation in hematological cancers are necessary.

Of note, there are also studies on site-specific *O*-GlcNAcylation in proteins that interact with NF-κB. It has been reported that NF-κB can be positively and negatively regulated by STAT5. The binding of NF-κB p65 to the IL-6 promoter is enhanced by STAT5 interaction in myeloid leukemic M1 cells (Kawashima et al., 2001). Interestingly, STAT5 *O*-GlcNAcylation was found to enhance its tyrosine phosphorylation to promote neoplastic myeloid transformation (Freund et al., 2017). However, STAT5 also competes with NF-κB for binding to target genes in B cell acute lymphoblastic leukemia (Katerndahl et al., 2017). How these interactions directly modulate STAT5-dependent NF-κB function remains to be determined.

## Crosstalk Between *O*-Glcnacylation and Other Posttranslational Modifications of Nuclear Factor-Kappab

The complexity and the diverse functional roles of *O*-GlcNAcylation, and its crosstalk with other PTMs of NF-κB [reviewed elsewhere (Perkins, 2006; Christian et al., 2016)], are immense. *O*-GlcNAcylation can act independently, directly compete with phosphorylation sites or modulate adjacent PTMs by altering the structure and/or binding properties of the protein. *O*-GlcNAcylation and phosphorylation often occur at the same or adjacent hydroxyl moieties. There has yet to be evidence to show competition between *O*-GlcNAcylation and phosphorylation at the same site in the five NF-κB subunits. Preliminary evidence suggests that p65 Thr-308 phosphorylation may impair Thr-305 *O*-GlcNAcylation (Ma et al., 2017). A similar crosstalk may also occur between phosphorylation sites at Ser-311 and Ser-316 phosphorylation of p65 and adjacent *O*-GlcNAcylation sites at Thr-305, Ser-319 or Ser-322 due to their proximity. *O*-GlcNAcylation can also negatively regulate p65 phosphorylation. Enhanced global *O*-GlcNAcylation following PUGNAc treatment, which also increases p65-specific *O*-GlcNAcylation, inhibits Ser-536 phosphorylation and NF-κB activation (Xing et al., 2011). In contrast, enhanced *O*-GlcNAcylation by OGT overexpression positively increases IKK-mediated Ser-536 phosphorylation of p65 contributing to NF-κB activation (Ma et al., 2017). Thus, it appears that an enhanced global *O*-GlcNAcylated state attained by OGA inhibition and an increase in *O*-GlcNAcylation cycling achieved by OGT overexpression yield contrasting outcomes, suggesting the need for careful choice in experimental methodology while studying *O*-GlcNAcylation. p65 *O*-GlcNAcylation at Thr-305 and Ser-319 has also been shown to enhance p65 acetylation at Lys-310 by p300 (Allison et al., 2012; Ma et al., 2017). OGT is essential for p300-mediated p65 Lys-310 acetylation (Allison et al., 2012), possibly through increasing p300 expression (Ma et al., 2017). p65 Lys-310 can also undergo methylation (Lu and Stark, 2015) although no studies have linked *O*-GlcNAcylation and methylation at this site (Figure 1). Much remains unknown on the mechanisms involved in this interplay, which may involve a plausible preferential recognition of *O*-GlcNAcylated p65 by p300 and formation of a p65, p300, and OGT complex.

Nominal information exists on the crosstalk between *O*-GlcNAcylation and other PTMs on other NF-κB pathway proteins (Figure 1). TAB3 *O*-GlcNAcylation at Ser-408 is required for its phosphorylation at Thr-404, which subsequently activates downstream TAK1 and NF-κB signaling. In contrast, the relationship between *O*-GlcNAcylation and phosphorylation in IKK2 appears to be competitive. Induction of *O*-GlcNAcylation of IKK2 at Ser-733 through glucose exposure, commonly found in oncogenic cells undergoing increased glycolysis, prevents the residue from functioning as an inactivating phosphorylation site thus creating a positive feedback loop to induce NF-κB activity (Kawauchi et al., 2009). Since IKK2 activity enhances cell viability in prostate cancer (Pflueger et al., 2011), *O*-GlcNAcylation of IKK2 may promote prostate cancer cell survival. Taken together, it appears that *O*-GlcNAcylation of upstream regulators of NF-κB pathway drives the NF-κB overactivity commonly seen in cancer.

## Proinflammatory Role of Nuclear Factor-Kappab *O*-Glcnacylation in Cancer

While the pathogenesis of cancer is varied, a common principle that underlies many tumorigenic processes is chronic inflammation. NF-κB is an important molecular link between inflammation and cancer. In hepatitis-associated neoplastic transformation, NF-κB activation enhances TNF-α, which in turn enhances NF-κB-dependent anti-apoptotic gene expression in a feed-forward loop (Pikarsky et al., 2004), and IKK2 is required for epithelial growth during colitis-associated cancer (Greten et al., 2004). There have been several reports suggesting the role of NF-κB *O*-GlcNAcylation in inflammation-induced cancer. Hyperglycemia-induced *O*-GlcNAcylation of p65 (Dela Justina et al., 2017) and c-Rel (Ramakrishnan et al., 2013) augments the production of inflammatory cytokines. Thr-322 *O*-GlcNAcylation of p65 has been proposed to control constitutive NF-κB activity in states of hyperglycemia (Yang et al., 2008). OGT-mediated *O*-GlcNAcylation of p65 and IKK1 promotes TNF-α and nitric oxide production in rat pancreatic acinar cells and progresses acute pancreatitis (Zhang et al., 2015). p65 *O*-GlcNAcylation at Thr-322 and Thr-352 also enhances DNA binding to the promoters of IL-6, TNF-α, and MCP1 which contributes to the development of colitis and colitis-associated cancer (Yang et al., 2015). Similar to p65, c-Rel Ser-350 *O*-GlcNAcylation may also contribute to an inflammatory state under hyperglycemic conditions via the expression of TCR-induced, CD28RE-dependent genes such as IL-2, CSF2, and IFNG (Ramakrishnan et al., 2013). Thus, c-Rel *O*-GlcNAcylation may contribute to inflammation-induced cancer or cancer-associated inflammation, both of which involve malignant cells utilizing excess glucose. Interestingly, c-Rel *O*-GlcNAcylation suppresses FOXP3 expression needed for the development of immunosuppressive Treg cells (de Jesus et al., 2021). Thus, c-Rel *O*-GlcNAcylation may also impart antitumor effects, as compromised Treg cell function may allow for improved cancer cell elimination by cytotoxic T cells. Further linking proinflammatory functions of NF-κB, *O*-GlcNAcylation and cancer, Ser-395 *O*-GlcNAcylation of TAB1 is required for NF-κB activation and expression of IL-6 and TNF-α (Pathak et al., 2012). Taken together, it appears that *O*-GlcNAcylation-dependent NF-κB functions may predominantly create a proinflammatory state to promote cancer development.

Mechanistic knowledge on the regulation of NF-κB by *O*-GlcNAcylation is limited. p65 *O*-GlcNAcylation decreases the binding of p65 to the inhibitor, IκBα, which increases p65 nuclear translocation and transactivation of proinflammatory genes (Yang et al., 2008). Whether c-Rel *O*-GlcNAcylation exerts a similar effect on IκBα is unknown. The mechanistic role of c-Rel *O*-GlcNAcylation has been implicated in the regulation of both protein-DNA and protein-protein interactions. *O*-GlcNAcylation regulates c-Rel-DNA binding and transcriptional activity both positively (Hwang et al., 2013; Ramakrishnan et al., 2013) and negatively (de Jesus et al., 2021). In addition, enhanced c-Rel *O*-GlcNAcylation following proinflammatory LPS treatment promotes interaction of c-Rel with p50 in microglia cells (Hwang et al., 2013) and *O*-GlcNAcylated c-Rel exists in complex with p65 in lymphocytes (Ramakrishnan et al., 2013). This indicates the intriguing possibility of a cell type specific *O*-GlcNAcylation-dependent NF-κB dimerization, which is an interesting future research direction.

## Anti-Inflammatory Role of Nuclear Factor-Kappab *O*-Glcnacylation in Cancer

A number of studies have found that NF-κB *O*-GlcNAcylation has an anti-inflammatory role. p65 *O*-GlcNAcylation was found to protect against inflammatory stress by attenuating NF-κB signaling in smooth muscle cells (Xing et al., 2011) and primary cultured cardiomyocytes (Zou et al., 2009). These findings were supported by the observations that glucosamine treatment improved cardiac function and attenuated inflammation following trauma hemorrhage or arterial damage and suppressed LPS-induced inflammation by reducing the amount of c-Rel *O*-GlcNAcylation and decreasing the production of inflammatory cytokines (Hwang et al., 2013). This countered many previous reports, which stated that increased concentrations of glucosamine would augment *O*-GlcNAcylation through the influx of the HBP pathway. While it is possible that the amount of *O*-GlcNAcylation enhancement after glucosamine treatment is indeed protein specific, it was later reported that the ability of glucosamine to impact c-Rel *O*-GlcNAcylation was dependent on glucose concentration in the culture conditions (Hwang et al., 2017). As these findings were in non-tumorous cells, it is possible that the context in which NF-κB is *O*-GlcNAcylated dictates its proinflammatory or anti-inflammatory capabilities. However, a later study showed that enhanced *O*-GlcNAcylation leads to a decrease in incidence and severity of inflammation-mediated colon carcinogenesis by suppressing NF-κB p65 phosphorylation and activation (Hirata et al., 2018). This directly opposes the results from Yang et al. (2015), which stated that enhanced p65 *O*-GlcNAcylation induces an inflammatory state and promotes colitis-associated cancer. These contrasting data may potentially be explained through their usage of differing mouse models. Yang et al., utilized an *Oga*^+/–^ mouse model to enhance *O*-GlcNAcylation while Hirata et al., implemented an *Ogt*-transgenic mouse. OGA has been reported to have histone acetylation activity (Toleman et al., 2004; Hayakawa et al., 2013) and partial deficiency of this protein may thus inadvertently decrease histone acetylation. OGT also interacts with multiple proteins, and its overexpression can lead to non-specific *O*-GlcNAcylation of cellular proteins. As such, these studies suggest and intricate relationship of glucose, glucosamine, inflammation, and warrants comprehensive studies on the specific role of *O*-GlcNAcylation in the context of cancer to derive mechanistic insights.

## Therapeutic Implications and Future Perspectives

Usage of NF-κB inhibitors to improve cancer therapy has long been discussed. Bortezomib, a first-in-class proteasome inhibitor with pan-NF-κB inhibitory function, has shown strong antitumor activity in multiple myeloma (Field-Smith et al., 2006) and AML (Attar et al., 2008; Colado et al., 2008; Howard et al., 2013), as well as in solid tumors such as preclinical models of breast (Teicher et al., 1999) and prostate (Adams et al., 1999) cancer. NF-κB inhibition using a non-degradable IκB super repressor (Duffey et al., 1999; Cusack et al., 2000; Arlt et al., 2002) or parthenolide (Sohma et al., 2011; Carlisi et al., 2017; Darwish et al., 2019) have been successful in various models. However, severe adverse effects have significantly hampered the clinical use of pan-NF-κB inhibitors due to the multifarious biological roles of NF-κB. This indicates a need for less toxic but still potent NF-κB inhibitors. Targeting specific PTMs of NF-κB could thus prove to be an ideal approach to target aberrant NF-κB functions in cancer while still maintaining its beneficial functions. Hence, the implications of an NF-κB-specific *O*-GlcNAcylation inhibitor are extremely promising with the potential to allow for optimal drug translation, but remains as an unmet need. As discussed previously, multiple *O*-GlcNAcylation sites have been identified in p65, with Thr-352 specifically required for its transcriptional activity (Yang et al., 2008). Inhibition of p65 *O*-GlcNAcylation at Thr-352 would likely dampen NF-κB overactivity and curtail the overexpression of p65-dependent genes, particularly those involved in tumor metastasis. However, the function of p65 *O*-GlcNAcylation has been found to both increase p65 DNA binding, as well as inhibit NF-κB activation. Taking into consideration NF-κB’s ability to act as both a tumor promoter and suppressor – as a word of caution - it is possible that enhanced p65 *O*-GlcNAcylation may upregulate or downregulate genes controlling cell proliferation or inflammation in a context dependent manner. c-Rel is only *O*-GlcNAcylated at Ser-350 (Ramakrishnan et al., 2013). c-Rel activity has been positively correlated with worse outcomes in hematological and solid tumors (Hunter et al., 2016). We have shown that *O*-GlcNAc modification of Ser-350 positively and negatively regulates c-Rel-dependent transcription (Ramakrishnan et al., 2013; de Jesus et al., 2021), and thus pharmacological regulation of Ser-350 in c-Rel could have significant benefits in both cancer and autoimmune disorders.

Current known roles of NF-κB *O*-GlcNAcylation are far from complete. Existing knowledge provides only partial insight on the role of *O*-GlcNAcylation in controlling p65 and c-Rel functions. Among the large number of upstream proteins regulating the NF-κB pathway, only three (IKK2, TAB1, and TAB3) have had their specific *O*-GlcNAcylation sites mapped (Table 1). Thus, identification of *O*-GlcNAcylation sites and function in other NF-κB subunits, (p105/p50, p100/p52, and RelB), and other key proteins regulating the canonical and non-canonical NF-κB pathways is an immediate need to be addressed in the field. Mechanistic knowledge gained through studying the regulation of NF-κB family of proteins by *O*-GlcNAcylation will have broad implications in learning how *O*-GlcNAcylation may control the functions of thousands of downstream proteins involved in carcinogenesis. Understanding the role of site-specific *O*-GlcNAcylation is essential in developing NF-κB PTM-specific cancer therapeutics that may exhibit relatively lower side effects than targeting total NF-κB proteins. Such novel therapeutics targeting *O*-GlcNAcylated NF-κB may position them as independent agents or as complements to current therapeutic regimens.

## Author Contributions

PR conceptualized the idea. AL wrote the manuscript. PR and AL edited, contributed to the article, and approved the submitted version.

## Conflict of Interest

The authors declare that the research was conducted in the absence of any commercial or financial relationships that could be construed as a potential conflict of interest.

## Publisher’s Note

All claims expressed in this article are solely those of the authors and do not necessarily represent those of their affiliated organizations, or those of the publisher, the editors and the reviewers. Any product that may be evaluated in this article, or claim that may be made by its manufacturer, is not guaranteed or endorsed by the publisher.
